# Human Umbilical Cord Mesenchymal Stem Cell-Derived Conditioned Medium Promotes Human Endometrial Cell Proliferation through Wnt/*β*-Catenin Signaling

**DOI:** 10.1155/2022/8796093

**Published:** 2022-08-30

**Authors:** Xiaoning Wei, Feiran Liu, Sichen Zhang, Xinyu Xu, Jin Li, Qingyu Wang, Jianping Cai, Shaowei Wang

**Affiliations:** ^1^Department of Gynecology and Obstetrics, Beijing Hospital, National Center of Gerontology, Institute of Geriatric Medicine, Chinese Academy of Medical Sciences, Beijing, China; ^2^Graduate School of Peking Union Medical College, Beijing, China; ^3^Department of Gynecology and Obstetrics, The First Affiliated Hospital of Guangxi Medical University, Nanning, Guangxi, China; ^4^Department of Obstetrics and Gynecology, Beijing Shijitan Hospital, Capital Medical University, Beijing, China; ^5^The Key Laboratory of Geriatrics, Beijing Institute of Geriatrics, Beijing Hospital, National Center of Gerontology, National Health Commission; Institute of Geriatric Medicine, Chinese Academy of Medical Sciences, Beijing, China

## Abstract

**Purpose:**

Mesenchymal stem cells (MSCs) and their derivant are among the promising treatments for intrauterine adhesion (IUA); they have been reported to repair the endometrial injury by proliferating endometrial cells. However, the signal pathways involved are not clear. This study investigated the role of human umbilical cord mesenchymal stem cell-derived conditioned medium (hUCMSC-CM) in relieving IUA to find out whether Wnt/*β*-catenin signaling was involved, and if so, to determine the possible ligands.

**Methods:**

After endometrial epithelial cells (EECs) were treated with hUCMSC-CM, their proliferation and migration were measured by the CCK8 assay and the scratch assay. The activation of Wnt/*β*-catenin signaling was measured by Western blots, fluorescent staining, and T-cell factor/lymphoid enhancer factor (TCF/LEF) luciferase. A Wnt inhibitor (XAV393) was used to inhibit the proliferation effect of hUCMSC-CM in EECs. Wnt5a expression in hUCMSC was measured by Western blots and fluorescent staining, and Wnt5a in hUCMSC-CM was detected by enzyme-linked immunosorbent assay (ELISA), to further clarify the mechanism.

**Results:**

As shown by the CCK8 assay, hUCMSC-CM promoted proliferation and migration of EECs. The expression of *β*-catenin, c-myc, and cyclin D1 increased in EECs after being treated with hUCMSC-CM. Moreover, hUCMSC-CM was found to promote *β*-catenin delivery into nuclei by Western blot and fluorescent staining; meanwhile, the inhibitor (XAV393) could restrain this process and inhibit the effect of hUCMSC-CM on EEC proliferation. Wnt5a was detected in hUCMSCs and hUCMSC-CM, which might be a potential therapeutic target.

**Conclusion:**

This study demonstrated that hUCMSC-CM promoted human endometrial cell proliferation through Wnt/*β*-catenin signaling, and Wnt5a might be a potential activator. This would be one of the activating signal pathways in the MSC-related treatment of IUA.

## 1. Introduction

Intrauterine adhesion (IUA), also known as Asherman's syndrome (AS), is a complex gynecological pathology mainly caused by the intrauterine operation, infection, and congenital anomaly of the uterus. It can be characterized by fibrous, connective tissue bands in the uterine cavity, with or without glandular tissue [1], leading to hypomenorrhea or amenorrhea, repeated pregnancy loss, and infertility [2]. Hysteroscopy is the first-line diagnostic investigation, and hysteroscopic adhesiolysis combined with hormone therapy had been used. However, with a high rate of recurrence after adhesiolysis [2], a new treatment was still being investigated. Human umbilical cord mesenchymal stem cell (hUCMSCs) transplantation was reported to repair the endometrial injury by proliferating endometrial cells [3]. Stem cell transplantation might be a potential treatment for IUA, but the tumorigenicity remained a problem since stem cell had the self-renewal capacity and multiple differentiation potentials. Recently, the conditioned medium (CM) of mesenchymal stem cells (MSCs) was shown to have a therapeutic potential similar to that of MSCs, which were repairing injured endometrium and restoring fertility, indicating that MSC-based therapy could be achieved through paracrine secretion [1]. Many cytokines were detected in MSC-CM [4], which is cell-free and rich in secreted bioactive factors, including a variety of protein, peptide, RNA, and lipid mediators [4]. It was still unclear which one played key role in IUA repairing.

Wnt5a/*β*-catenin signaling is critical in estrogen-mediated uterine development [5]. It can be induced by estradiol [6], participating in the development and functional maintenance of the endometrium [7, 8] and modulating the self-renewal activity of endometrial mesenchymal stem cells (eMSCs) [9–11], indicating that it might be a potential target in IUA treatment. Wnt ligands were found in hUCMSC-derived exosomes [12], promoting *β*-catenin nuclear translocation and enhancing the proliferation of skin cells. Wnt5a could also be secreted and transported in extracellular vesicles [13].

In this study, we investigated the role of hUCMSC-CM in promoting the proliferation and migration of endometrial epithelial cells (EECs) to find out whether Wnt5a derived from hUCMSC-CM could activate *β*-catenin signaling in endometrial cells.

## 2. Methods

### 2.1. Ethics Statement

For this study, hUCMSCs were isolated from umbilical cords acquired from the Department of Obstetrics of Beijing Hospital, according to the protocol approved by the Ethics Committee of Beijing Hospital (no. [2019]04). The donors also provided informed consent, in accordance with the Declaration of Helsinki. Human EECs were purchased from Procell Life Science & Technology Co., Ltd., Wuhan, China. The authors had no conflict of interest.

### 2.2. Isolation and Characterization of Human Umbilical Cord Mesenchymal Stem Cells (hUCMSCs)

The umbilical cords were washed with phosphate buffer saline (PBS, 0.1 M, pH 7.4) containing 5% penicillin/streptomycin (P/S). Wharton's jelly was cut into small pieces and exposed to collagenase type IV solution (1 : 1 in PBS) for 1 h. They were cultured in Dulbecco's modified Eagle's medium (DMEM/F12, Gibco, Hyclone), supplemented with 10% fetal bovine serum (Gibico) and 1% P/S, and incubated in a humidified atmosphere containing 5% CO_2_ at 37°C. The medium was changed every day. Next, the large particle pieces were removed, and the adherent cells were subcultured using 0.25% trypsin. The hUCMSCs from the third to the fifth passages were used for further experiments [14].

The hUCMSCs were verified by a flow cytometer (Beckman Coulter, Brea, CA, USA) after staining with the specific antibodies, including CD 34, 44, 45, 73, 90, and 11b conjugated with FITC and APC, respectively.

### 2.3. Preparation of hUCMSC-CM

The hUCMSCs (third passage) were washed with PBS three times until they were 70–80% confluent, then they were preincubated with serum-free fresh DMEM/F12 for 48 h. The CM was collected, centrifuged at 1,000 rpm for 20 min, and filtered through a 0.22 um filter.

### 2.4. ELISA

Wnt5a in the CMs was measured by the enzyme-linked immunosorbent assay (ELISA) according to the manufacturer's instructions (MLBio, Shanghai, China).

### 2.5. Proliferation Assay

EECs (P3) were seeded in 96-well plates (1 × 10^4^ cells/well) after being cultured with hUCMSC-CM or serum-free DMEM/F12 for 48 h. The CCK-8 reagent (10 *μ*l; Beyotime, Jiangsu, China) was then added to the plates, which were incubated in a humidified atmosphere containing 5% CO_2_ at 37°C for 3 hours, and each sample was measured at 450 nm.

### 2.6. mRNA Isolation, cDNA Synthesis, and Real-Time RT-PCR

EECs were pretreated with hUCMSC-CM or serum-free MDEM/F12 in 6 cm plates for 48 h. The cells were collected, and the total RNA was extracted by an RNA isolation kit (Vazyme, Nanjing, Jiangsu Province, China), followed by a reverse transcription using a cDNA synthesis kit (TransGen Biotech, Beijing, China). The cDNA was followed by a real-time quantitative polymerase chain reaction (PCR) using the KAPA SYBR® FAST Master Mix (KAPA BIO, Boston, MA, USA) with a primer. Each gene expression level was normalized, with GAPDH used as a housekeeping control. The primer sequences were as follows: Wnt5a, forward 5′-CTCGCCATGAAGAAGTCCA-3′ and reverse 5′- TACCTAGCGACCACCAAGAA -3′; cyclin D1, forward 5′- GCTGCGAAGTGGAAACCATC -3′ and reverse 5′- CCTCCTTCTGCACACATTTGAA -3′; c-myc, forward 5′- GTCAAGAGGCGAACACACAAC -3′ and reverse 5′- TTGGACGGACAGGATGTATGC -3′; CTNNB1, 5′- GGTGGGCTGCAGAAAATGGTT -3′ and reverse 5′- GATGGCAGGCTCAGTGATGTCTTC -3′.

### 2.7. Western Blotting

Cells were lysed with RIPA lysis buffer (Solarbio, Beijing, China) containing 1 × PMSF (Solarbio, Beijing, China) to extract total protein.

Nuclear and cytoplasmic proteins were extracted separately with the Nuclear and Cytoplasmic Protein Extraction Kit (Beyotime, Jiangsu, China). Protein lysates (20 *μ*g) were separated by 12% sodium dodecyl sulfate-polyacrylamide gel electrophoresis (SDS-PAGE) and transferred to polyvinylidene fluoride (PVDF) membranes (0.45 *μ*m; Millipore, Burlington, MA, USA). The membranes were incubated with antibodies against *β*–catenin (1 : 4000 in antibody dilution buffer (Beyotime, Jiangsu, China), the following antibodies used the same dilution buffer), C-myc (1 : 1000), Cyclin D1(1 : 1000), GAPDH (1 : 5000), Wnt5a (1 : 1000), *β*-tubulin (1 : 2000) (Abcam, Cambridge, UK), and Histone (1 : 2000) (Cell Signaling Technology, Danvers, MA, USA) at 4°C overnight and then incubated with corresponding horseradish peroxidase- (HRP-) conjugated second antibodies (1 : 1000) (Cell Signaling Technology, Danvers, MA, USA) at 37°C for 1 h. The bands were visualized with enhanced chemiluminescence (Millipore, Burlington, MA, USA). The intensity of each band was calculated using Image J software (National Institutes of Health, MD, USA).

### 2.8. Immunofluorescence Staining

After treatment, the cells were fixed in 4% paraformaldehyde, permeabilized with 0.3% Triton X-100 in PBS, and blocked in 1% bovine serum albumin for 1 h. Then, the cells were incubated with primary *β*-catenin antibodies (1 : 200) (Abcam, Cambridge, UK) at 4°C overnight in a humidified atmosphere. They were then incubated with Alexa Fluor488-conjugated secondary antibodies (1 : 500) (Proteintech, Chicago, IL, USA) for 1 h, and the nucleus was stained with DAPI (Beyotime, Jiangsu, China) for 5 min. Immunofluorescence staining was imaged using fluorescence microscopy (Cannon, Tokyo, Japan).

### 2.9. TOP/FOP Luciferase Reporter Assay

The cells were seeded into a 24-well plate at a density of 50,000 cells per well. The cells were cotransfected with 0.5 *μ*g of either TOPflash or FOPflash vector (Beyotime, Jiangsu, China) and 0.1 *μ*g of pRL-TK (Renilla-TK-luciferase vector) as a control using Lipofectamine 3000 (Invitrogen). Some cells were subsequently treated with hUCMSC-CM, while the control group was treated with the serum-free DMEM/F12 for 48 h. The cells were then lysed, and the luciferase activities were measured using the Dual-Luciferase Reporter Gene Assay Kit (Beyotime, Jiangsu, China), according to the manufacturer's instructions. Firefly luciferase activity was normalized against the Renilla luciferase activity, and the TOP/FOP ratio was used as a measure to evaluate the activation of the T-cell factor/lymphoid enhancer factor (TCF/LEF) transcription.

### 2.10. Scratch Assay

The cells were seeded in 6-well plates at 5 × 10^5^ cells per well. After cell adherence, scratches were made with a sterilized P200 pipette tip (500-*μ*m width), and the cells were cultured in hUCMSC-CM or serum-free DMEM/F12 after washing with PBS. After 0 h, 48 h, and 96 h, the scratches were photographed by microscopy (Canon, Tokyo, Japan) and measured manually with Image J software. The data were reported as the ratio of migration relative to the control.

### 2.11. Statistics

The results are expressed as mean ± SEM. All experiments were repeated three times with independent cultures. Statistical significance was assessed using Student's *t*-test, and a *P* value < 0.05 indicated significant differences.

## 3. Results

### 3.1. Characterization of hUCMSCs

Flow cytometry was used to detect the positive markers (CD44, CD73, and CD90) and the negative markers (CD45, CD34, and CD11b) of the MSCs to identify the hUCMSCs. The results demonstrated that the positive markers were highly expressed, but the negative markers were not expressed (Figure 1).

### 3.2. hUCMSC-CM Promoted the Proliferation and Migration of Endometrial Cells

The CCK8 assay was performed to investigate the effect of hUCMSC-CM on endometrial cells proliferation. The results showed that hUCMSC-CM promoted the proliferation of EECs (Figure 2(a)). The scratch assay showed that hUCMSC-CM enhanced the EECs' migration property compared with the control group (Figure 2(b)).

### 3.3. hUCMSC-CM Activated Wnt/*β*-Catenin Pathway of Endometrial Cells In Vitro

After being treated with hUCMSC-CM for 48 h, the mRNA expression of CTNNB1 in EECs was detected. The results of the CTNNB1 gene expression were significantly higher in the hUCMSC-CM group than in the control group (treated with serum-free DMEM/F12) (Figure 3(a)), and the results were confirmed (by Western blotting) in the protein levels (Figure 3(b)).

After being treated with hUCMSC-CM for 48 h, the mRNA expression of downstream gene CMYC and CYCLIND1 in EECs was detected. The CYCLIND1 gene expression was significantly higher in the hUCMSC-CM group than that in the control group (treated with serum-free DMEM/F12), while C-MYC showed no statistical difference (Figure 3(a)). Both had no statistical difference in protein levels (Figure 3(b)).

Furthermore, the *β*-catenin protein levels in nucleus and cytoplasm were detected, respectively. In the hUCMSC-CM groups, the *β*-catenin protein levels were higher in nucleus than those of the control groups (Figure 3(d)), and they showed nuclei located in immunofluorescence staining (Figure 3(c)). TCF/LEF luciferase activities were measured in these two groups. The results showed that hUCMSC-CM increased the TCF/LEF luciferase activities of endometrial cells (Figure 3(e)), indicating that hUCMSC-CM can promote nuclear localization of *β*-catenin and transcriptional activation of the Wnt/*β*-catenin pathway in EECs in vitro.

### 3.4. Wnt5a Expression in hUCMSCs and hUCMSC-CM

To explore which protein might activate the Wnt/*β*-catenin in endometrial cells, the expression of Wnt5a in hUCMSCs was confirmed by Western blotting. The protein expression levels of Wnt5a were significantly higher in hUCMSCs than that in EECs (Figure 4(a)). By immunofluorescence staining, we also detected the Wnt5a protein located in the plasma of hUCMSCs (Figure 4(b)). By ELISA, we detected the concentration of Wnt5a in the culture supernatant (Figure 4(c)). The results showed that the level of secreted Wnt5a was higher than that in the control group (serum-free DMEM/F12). This data showed that Wnt5a was produced by hUCMSCs and secreted into hUCMSC-CM.

### 3.5. XAV939 Inhibited the Proliferation Effect of hUCMSC-CM in Endometrial Cells

Loss-of-function approaches were used to assess the role of Wnt/*β*-catenin signaling in the proliferation of endometrial cells. XAV939 is a potent tankyrase inhibitor that targets Wnt/*β*-catenin signaling, stabilizing axin, thereby stimulating *β*-catenin degradation. The addition of XAV939 (at a concentration of 50 *μ*mol/ml) to hUCMSC-CM inhibited the proliferation of endometrial cells in the control group compared with the hUCMSC-CM group (Figure 5(a)). Being degraded, *β*-catenin protein delivered into nuclei would also be inhibited (Figure 5(b)).

## 4. Discussion

In this study, we explored the effect of hUCMSC-CM on promoting human endometrial cell proliferation and found that Wnt/*β*-catenin signaling was activated in this process. Our results showed that hUCMSC-CM could activate Wnt/*β*-catenin signaling in promoting EECs proliferation; meanwhile, by inhibiting the signaling, the proliferation of EECs was restrained. We also found that the signaling was probably activated by Wnt5a secreted by hUCMSCs, which was detected in the cytoplasm, and also in the hUCMSC-CM.

Recently, there have been several studies on stem cells therapy in IUA in animals and human beings. Bone marrow stem cell intrauterine transplantation can improve the fertility outcome in IUA mice [15]. The therapeutic effect of MSCs had been verified in IUA patients [16, 17]. As we know, the endometrium of the uterus has a regenerative capacity. During each menstrual cycle, it undergoes a process of degeneration, proliferation, differentiation, and regeneration. Stem cells were believed to reside in the basal layer of the endometrium [18, 19]. When the uterine injury occurred, stem cells were recruited and differentiated to repair the impairment, likely due to immunomodulation, recruitment of growth factors, and paracrine effects [2]. In our previous study, MSCs secreted a multitude of cytokines and signaling molecules that promote the endometrial proliferation and glandular reformation after trauma, including epidermal growth factor (EGF), insulin-like growth factor-binding protein (IGFBP), insulin-like growth factor-1 (IGF-1), and fibroblast growth factor (FGF) [20]. MSC-CM contained a variety of protein, peptide, RNA, and lipid mediators [4], also shown to have a therapeutic effect on IUA as in the case of stem cells. However, the mechanisms and signaling pathways involved remained unclear.

The Wnt signaling pathway is an essential cellular signaling pathway in organisms, which often involves in embryonic development and cell proliferation [21]. This pathway can be divided into two forms: the canonical and the noncanonical types. The noncanonical pathway includes the noncanonical planar cell polarity (PCP) pathway and the Wnt/calcium pathway.

In the canonical Wnt signaling pathway, also known as the Wnt/*β*-catenin pathway, Wnt ligands bind to the frizzled (Fzd) receptor and coreceptor and low-density lipoprotein receptor-related protein 5/6 (LRP 5/6), initiating *β*-catenin nuclear translocation. *β*-Catenin is an unstable protein and is strictly regulated in the cytoplasm. In the absence of a Wnt ligand, intracellular *β*-catenin is targeted by a degradation complex. The complex consists of tumor suppressor protein (APC), scaffold protein Axin, and two kinases: tyrosine kinase 1*α* (CK1*α*) and glycogen synthase kinase 3*β* (GSK-3*β*). CK1*α* and GSK-3*β* phosphorylated *β*-catenin N-terminal serine and threonine, phosphorylated *β*-catenin recognized by transducers, which are part of the ubiquitin ligase complex, then *β*-catenin was degraded after ubiquitination. When the Wnt ligand binds to Fzd and LRP5/6, it induces phosphorylation of disheveled protein (DVL/DSH), recruits Axin protein, and then disintegrates the degradation complex. *β*-Catenin accumulates in the cytoplasm and translocates into the nucleus, where it binds to the TCF/LEF to regulate the target gene of the Wnt pathway [21].

The canonical Wnt signaling pathway plays a role in endometrial cell proliferation. Nei and his colleagues [22] collected the normal endometrial tissue, endometrial hyperplasia tissue, and endometrial cancer. They found that *β*-catenin was expressed in endometrial tissue in the middle and the late proliferation phases and increased in the nucleus of proliferative endometrial cells stimulated with high-dose estrogen without progesterone. In the secretion phase, when progesterone increases and estrogen decreases, the nucleus *β*-catenin decreases. Hou et al. [23] detected *β*-catenin in the nucleus of the endometrial epithelium after giving exogenous estrogen to mice. Furthermore, they delivered adenoviral expressed SFRP2, the Wnt signaling inhibitor, in mice and observed that estrogen-induced promotion of EECs proliferation was inhibited. Gunin et al. [24] inhibited GSK3*β* by giving LiCl, activator of the Wnt/*β*-catenin pathway, and successfully simulated the proliferation of endometrium in mice.

Wnt signaling molecules can also activate eMSCs and participate in endometrial periodic regeneration. Cao et al. [9] found that coculture of myometrial cells enhanced the colony forming and self-renewal ability of eMSCs. It is believed that Wnt/*β*-catenin signaling was involved. By using the Wnt pathway activator (Wnt3a CM) and the Wnt inhibitor (XAV939 and IWP-2), the participation of *β*-catenin signaling in the self-renewal of eMSCs was confirmed. The high expression of Wnt5a was detected in uterine myocytes. The introduction of recombinant Wnt5a can stimulate eMSCs colony formation, while the Wnt5a antibody inhibited the colony formation. It is inferred that uterine myocytes are the activated microenvironment components of eMSCs, and the Wnt5a/*β*-catenin signaling pathway is an important signaling pathway to activate eMSCs. Bukowska et al. [25] found that the inhibitor (XAV939) and the activator (BIO) of the canonical Wnt signaling pathway could upregulate and downregulate the stem cell markers (CD73 and CD105), respectively, indicating that the activation of the canonical Wnt signaling pathway led to the differentiation of eMSCs.

C-myc and cyclin D1 are the downstream genes of Wnt/*β*-catenin signaling [26, 27]; they are also estrogen-regulated genes implicated in cell proliferation. C-myc is a proto-oncogene, which had been reported to encode a transcriptional regulatory protein required for cell growth [28] and modulate the expression of cyclin D1, a cell cycle control gene [29]. It can be upregulated by estrogen and found increased expression in endometriosis [30]. In this study, they were upregulated by hUCMSC-CM along with *β*-catenin, indicating that the component in the hUCMSC-CM might activate Wnt/*β*-catenin signaling, upregulate the expression of c-myc, and regulate the cell cycle of EECs, promoting the cells' proliferation.

Many proteins are responsible for the development and regeneration of the endometrium, of which Wnt, c-kit (CD117), Oct-4, CD34/KLF4, and Musashi-1 are the best classified [2]. In this study, Wnt/*β*-catenin signaling was activated by hUCMSC-CM, participating in EEC proliferation. Wnt genes were found expressed in hUCMSCs; among them, a relatively high mRNA expression of the Wnt5a was detected [31]. Consistent with our results, the Wnt5a protein was found expressed in hUCMSCs and enriched in hUCMSC-CM, indicating that Wnt5a/*β*-catenin signaling might be involved.

## 5. Limitations

Regarding the limitations of our work, first, the complex signal network and cross-talk are not discussed in this article. Second, other Wnt-ligand proteins, such as Wnt7a and Wnt4, were reported to play an essential role in endometrial development and regeneration of reproductive tracts; however, whether or not they relate to IUA treatment has not been addressed in this paper. Third, the Wnt/*β*-catenin pathway has been examined in vitro; in vivo studies need to be conducted in future work.

## 6. Conclusion

Our study demonstrated that hUCMSC-CM promoted human endometrial cell proliferation through Wnt/*β*-catenin signaling, and Wnt5a might be an activator. This would be one of the activating signal pathways in the MSC-related therapy of IUA.

## Figures and Tables

**Figure 1:** Characterization of MSCs. Flow cytometry analysis of common MSC markers such as (a) CD44, (b) CD73, and (c) CD90. MSCs are negative for (d) CD45, (e) CD34, and (f) CD11b.

**Figure 2:** Cell proliferation and migration activity of EECs treated with hUCMSC-CM. (a) Cell proliferation of EECs with serum-free DMEM/F12 (control group) or hUCMSC-CM (experimental group). (b) The image of cell migration of EECs cultured with serum-free DMEM/F12 (control group) or hUCMSC-CM. Scale bar: 20 *μ*m. ^∗∗∗^*P* < 0.001.

**Figure 3:** hUCMSC-CM activated Wnt/catenin signaling pathway. (a) CTNNB1, CMYC, and CYCLIND1 gene expressions were measured by RT-PCR in EECs treated with serum-free DMEM/F12 (control group) or hUCMSC-CM. (b) Western blotting images and relative quantitative analysis of total *β*-catenin, c-myc, and cyclin D1 protein in EECs. EECs were treated with serum-free DMEM/F12 (control group) or hUCMSC-CM. (c) Immunofluorescence staining of *β*-catenin protein in EECs after serum-free DMEM/F12 (control group) or hUCMSC-CM treatments. Scale bar: 20 *μ*m. (d) Western blotting determined the nuclear and cytoplasmic *β*-catenin levels in EEC cells after serum-free DMEM/F12 (control group) or hUCMSC-CM treatments. (e) The TCF/LEF luciferase signals in EECs after serum-free DMEM/F12 (control group) or hUCMSC-CM treatments. ^∗^*P* < 0.05; ^∗∗^*P* < 0.01.

**Figure 4:** Wnt5a expression in human MSCs. (a) Western blots of Wnt5a and corresponding semiquantitative analysis using EECs as control. (b) Immunofluorescence staining of Wnt5a in hUCMSCs. Scale bar: 10 *μ*m. (c) Wnt5a was quantified in the hUCMSC-CM by ELISA, with serum-free DMEM/F12 as control. ^∗∗∗^*P* < 0.001; ^∗∗∗∗^*P* < 0.0001.

**Figure 5:** The proliferation of endometrial cells treated with hUCMSC-CM is inhibited by XAV939. (a) The proliferation of EECs treated with serum-free DMEM/F12 + DMSO (control group), hUCMSC − CM + DMSO, and hUCMSC − CM + XAV939 (50 *μ*mol/ml). (b) Western blotting images and quantitative analysis of *β*-catenin protein levels in nucleus and cytoplasm ^∗^*P* < 0.05; ^∗∗∗^*P* < 0.001; ^∗∗∗∗^*P* < 0.0001.

## Data Availability

The data used to support the findings of this study are currently under embargo while the research findings are commercialized. Requests for data, 12 months after publication of this article, will be considered by the corresponding author.
